# Therapeutic Effect of Continuous Blood Purification Combined with Humanized Nursing in Patients with Severe Sepsis

**DOI:** 10.1155/2022/1411371

**Published:** 2022-08-16

**Authors:** Lili Gan, Jiafeng Hu, Li Xia, Xiaoqin Xi

**Affiliations:** Department of Blood Purification Centre, First People's Hospital of Linping District, Hangzhou 311100, Zhejiang, China

## Abstract

This work aimed to explore the effect of humanized nursing on the patients' recovery from severe sepsis based on continuous blood purification (CBP). 90 patients with severe sepsis were randomly and equally divided into a control group (basic intensive nursing + CBP) and a therapy group (humanized nursing + CBP). Before treatment and on the 7th and 14th days after treatment, indicators of patients were compared, including white blood cell (WBC), tumor necrosis factor (TNF-*α*), hepatic and renal function, C-reactive protein (CRP), brain natriuretic peptide (BNP), procalcitonin (PCT), and erythrocyte sedimentation rate (ESR). The mortality and nursing satisfaction were compared. After treatment, the saturation of pulse oxygen (SPO_2_) in the therapy group (85 ± 20 and 91 ± 9) was higher than that in the control group (78 ± 28 and 82 ± 18, respectively), and the lactic acid level (LAL) was greatly lower (2.8 ± 2.4 and 1.6 ± 0.9 vs. 4.3 ± 2.3 and 2.3 ± 2.7). The Acute Physiology and Chronic Health Evaluation II (APACHE-II) score after treatment was lower (13.67 ± 4.28 and 8.45 ± 5.12 vs. 17.34 ± 6.4 and 11.46 ± 4.23). The BNP, blood urea nitrogen (BUN), and CRP levels were decreased, and so did inflammatory indicators. The survival rate reached 71% and 47% in the therapy group and control group, respectively; and the nursing satisfaction was 97.80% and 26.67%, respectively. Humanized nursing combined with CBP could improve the therapeutic effect and speed up the recovery from severe sepsis.

## 1. Introduction

Sepsis is a systemic inflammatory response syndrome caused by severe infection, which often occurs in patients who have experienced severe burns, severe pneumonia, or extensive skin damage [1]. Inflammation caused by severe sepsis can lead to varying degrees of failure of the body's organ function or malfunction of the body's circulation. The common pathogenic bacteria that cause sepsis mainly include *Staphylococcus*, *Streptococcus*, *Enterococcus*, Gram-negative bacilli, and fungi [2]. Typical sepsis patients may experience chills, high fever, general malaise, headache, joint pain, fatigue, rapid pulse, and shortness of breath. Peripheral blood examination showed significantly increased white blood cells (WBC), usually up to (10–30) × 10^9^/L; specifically, neutrophils were significantly increased, and there were obviously left-shifted nuclei in intracellular toxic granules. The clinical diagnosis of sepsis is mainly based on blood or bone marrow culture results [3, 4]. The infection caused by sepsis will involve multiple organs, leading to the failure of multiple organs in the whole body. If not treated in time, it will cause severe sepsis and septic shock, and the mortality rate is high. In the intensive care unit, if a patient develops septic shock, the mortality rate can reach 30%∼80%. Therefore, patients should pay enough attention to the early manifestations of sepsis and receive timely treatment and intervention [5].

Continuous blood purification (CBP), also known as continuous renal replacement therapy (CRRT), is currently one of the main treatments for patients with sepsis [6]. It functionally replaces the kidneys of the human body, makes up for the decline or failure of the kidneys caused by sepsis, circulates the blood outside the body, and uses instruments to filter the blood. To a greater extent, it can purify the toxic substances in the blood and reduce the filtering pressure of the kidneys, thereby maintaining the body's metabolic function at a normal level [7]. In addition, CBP also provides better room for the recovery of the kidneys. However, CBP involves the extracorporeal circulation of blood. In this process, if the sterility of the operating environment cannot be guaranteed, or the equipment pipelines and filter connections are not tightly connected, the patient may be reinfected, aggravating the disease [8, 9]. During blood circulation, coagulation may also occur. Timely use of anticoagulants according to the patient's condition can effectively alleviate the coagulation situation, thereby ensuring the smoothness of vascular access and filters and reducing unnecessary medical expenses for patients. During CBP, it will not only filter out the toxic substances in the blood, but also remove some nutrients. At this time, giving appropriate nutritional support will help patients recover [10]. In addition, the vital signs of patients with severe sepsis are unstable. Controlling the treatment speed during CBP and monitoring the patient's heart rate and blood sugar can help to help the patient's disease treatment. The abovementioned measures applied to CBP can improve the therapeutic effect to a certain extent.

To sum up, this work innovatively included the abovementioned operations into the scope of humanized nursing in this experiment, and compared it with a conventional nursing intervention to judge the therapeutic effect of continuous blood purification combined with humanized nursing intervention, aiming to provide some theoretical support for clinical treatment of patients with severe sepsis and help their recovery.

## 2. Materials and Methods

### 2.1. General Data

In this work, 90 patients with severe sepsis who were admitted to First People's Hospital of Linping District from October 2021 to January 2022 were selected as the research objects. They were randomly divided into a control group and an observation group, with 45 cases in each group. There were 23 males and 22 females in the observation group, with an age distribution range of 32–73 years old and an average age of 44.25 ± 8.27 years old. The control group consisted of 22 males and 23 females, with an age distribution range of 30–75 years old and an average age of 43.75 ± 7.56 years old. There were no significant differences in age, gender, educational level, body mass index, and smoking history between the two groups of subjects (*P* > 0.05). The study has been approved by the Medical Ethics Committee of First People's Hospital of Linping District, and the patients and their families understood the research content and methods and agreed to sign the corresponding informed consent.

Inclusion criteria were given as follows: all newly admitted patients were clearly diagnosed with severe sepsis; patients combined with multiple organ failure; and patients whose condition information was detailed.

Exclusion criteria were given as follows: patients with AIDS, malignant tumor, endocrine disease, blood disease or immune-related disease, hormone, and immunosuppressive therapy, abandoned treatment, and incomplete case data; patients with sepsis who are seriously ill and not suitable to participate in this study; and patients with Acute Physiology and Chronic Health score (APACHE-II score) greater than 30 points.

### 2.2. Methods

On the basis of adequate antishock, anti-infection, and nutritional support treatment, continuous blood purification was performed on the two groups of patients. The specific operation of continuous blood purification was shown in Figure 1. Afterward, the control group was given routine nursing (guiding patients to rest in bed and reasonable diet), and the observation group was given humanized nursing intervention on the basis of the control group.

### 2.3. Humanized Nursing

Measures related to humanized nursing were summarized as follows: Firstly, mental health had to be cared for. The patient would have physical resistance or psychological resistance due to the torment of the disease, resulting in emotional instability. Psychological counseling was required, and it should actively be communicated with family members to meet the needs of the patient as much as possible. Secondly, it could educate the disease knowledge. In order to stabilize or accelerate the recovery of the disease, it is necessary to strengthen the health education of patients and their families and prepare corresponding health knowledge based on the specific situation of the patient, such as diet, precautions for work and rest, and knowledge of disease diagnosis and treatment [7]. Thirdly, it could strengthen the supervision of complications during patient treatment, including disinfection and isolation (regular ward disinfection and strict aseptic operation), anticoagulation prevention and care (heparin anticoagulation according to the situation), monitoring of volume balance (control of water, electrolytes, and pH balance), vascular access care (avoid blockage, bending, and regular cleaning), body temperature monitoring, and nutritional support [11, 12]. Finally, it should continuously monitor the electrocardiograph (ECG), regularly monitor blood electrolytes, hepatic and renal function, and blood gas analysis; maintain the balance of body water, electrolyte, and pH value; and detect the blood sugar to avoid symptoms such as hypokalemia and hypocalcemia [13].

### 2.4. Observation Indicators

Before the patients received the corresponding treatment and on the 7th and 14th days after the treatment, white blood cell (WBC), tumor necrosis factor (TNF-*α*), liver and kidney function, C-reactive protein (CRP), serum brain natriuretic peptide, procalcitonin (PCT), and erythrocyte sedimentation rate (ESR) were collected and analyzed. In addition, it should dynamically monitor the level of consciousness, vital signs, arterial blood gas analysis, and changes in lactate, and compare the APACHE-II score in different stages of treatment [14]. The mortality and survival rate of patients in the experimental stage were observed, the complications after nursing intervention were observed, and the patients' satisfaction with humanized nursing was collected. Nursing satisfaction took the final score of the questionnaire as the patient's score of nursing satisfaction. The total score was 100 points: very satisfied, above 90 points; satisfied, 60–90 points; average, below 60.

### 2.5. Experiment Process

The specific experiment process is illustrated in Figure 2.

### 2.6. Statistical Methods

SPSS 24.0 was adopted to analyze the obtained data, among which the measurement data was expressed as (*x* ± *s*) and was analyzed by *t*-test; while the count data was expressed as (%). The comparison between the two groups was performed by the chi-square test, and *P* < 0.05 meant the difference was statistically significant.

## 3. Results

### 3.1. General Data of Patients

Before treatment, body temperature, respiration, heart rate, SPO_2_, and lactate acid level (LAL) were measured, and it was found that there was no significant difference between the control group and the therapy group (*P* > 0.05). On the 7th and 14th days after receiving the treatment, the SPO_2_ (85 ± 20 and 91 ± 9, respectively) of the therapy group under the intervention of humanized nursing was significantly higher than that of the control group (78 ± 28 and 82 ± 18, respectively). In addition, the value of the therapy group on the 7th day was higher than that of the control group on the 14th day. The LAL (2.8 ± 2.4 and 1.6 ± 0.9, respectively) was significantly lower in contrast to the control group (4.3 ± 2.3 and 2.3 ± 2.7, respectively), and the decline rate was higher than that of the control group, showing statistically obvious differences (*P* < 0.05). The specific data results are given in Figure 3.

### 3.2. Comparison of APACHE-II Scores

There was no significant difference in APACHE-II score before receiving the corresponding treatment (*P* > 0.05). After treatment, the APACHE-II scores of the control group (17.34 ± 6.4, 11.46 ± 4.23) and the observation group (13.67 ± 4.28, 8.45 ± 5.12) were reduced to varying degrees on the 7th and 14th days. Compared with the control group, the scores on the 7th and 14th days in the observation group decreased significantly, and the final APACHE-II score also showed that the observation group was significantly smaller than the control group, and the difference was statistically significant (*P* < 0.05). Refer to Figure 4 for details.

### 3.3. Comparison of Routine Blood Biochemical Indicators

Before receiving treatment, the differences in serum brain natriuretic peptide, blood urea nitrogen, and creatinine between the observation group and the control group were not statistically significant (*P* > 0.05). After receiving treatment, the blood biochemical indexes of the two groups were decreased to varying degrees on the 7th day and the 14th day. However, compared with the control group, the observation group showed a more obvious downward trend, and the improvement of serum brain natriuretic peptide, blood urea nitrogen, and creatinine were more obvious, and the difference was statistically significant (*P* < 0.05). The specific contents are shown in Figure 5.

### 3.4. Comparison of Inflammatory Indicators

Before receiving treatment, there was no significant difference in inflammatory indicators (WBC, CRP, ESR, PCT, and TNF-*α*) of patients between the two groups (*P* > 0.05). On the 7th and 14th days after receiving treatment, the levels of WBC, CRP, ESR, and PCT in both groups all decreased (as demonstrated in Figure 6). Compared with the control group, those in the therapy group decreased more significantly, and the differences were statistically significant (*P* < 0.05).

### 3.5. Comparison of Immune Indicators

Before treatment, there were no significant differences in the levels of cellular immune indicators reflected by the corresponding T lymphocyte subsets of helper T cells CD4+, cytotoxic T cells CD8+, and the ratio of CD4+ to CD8+ (CD4+/CD8+) between the two groups of patients (*P* > 0.05). On the 7th and 14th days after treatment, the levels of CD4+ and CD4+/CD8+ in the therapy group and the control group showed an upward trend, and the difference was statistically significant (*P* < 0.05). In addition, the levels of CD8+ showed a significant decrease (*P* < 0.05). The CD8+ level, CD4+ level, and CD4+/CD8+ level of the therapy group were higher than those of the control group (*P* < 0.05), as shown in Figure 7.

### 3.6. Comparison of the Prognosis of the Two Groups of Patients

The prognosis of the patients in the observation group and the control group is shown in Table 1. The patient's survival rate, case fatality rate, and discontinuation of treatment for other reasons within 14 days of treatment were used as treatment endpoints. During this period, according to statistics, the survival rate of the observation group was as high as 71%, and the survival rate of the control group was 47% lower than that of the observation group. The observation group had a significant advantage, and the difference was statistically significant (*P* < 0.05). The mortality rate between the two groups was compared. It can be observed that the mortality rate of the observation group (24%) was also significantly lower than that of the control group (42%), and the difference was statistically significant (*P* < 0.05). With nursing intervention, the patient's acceptance of treatment is higher, and the treatment attitude is more positive. Therefore, the corresponding proportion of giving up treatment due to psychological and physical reasons was also less than 5%, and the difference was statistically significant (*P* < 0.05). The comparison of the three prognostic indicators is shown in Figure 8.

### 3.7. Incidence of Complications

Under the nursing intervention, the probability of complications for the patients was also greatly reduced. The probability of lactic acid accumulation, abnormal body temperature, pipeline blockage, and coagulation disorder in the observation group was only 4.4%, which was significantly lower than that in the control group (15.6%), and the difference was statistically significant (*P* < 0.05). The details are shown in Table 2:

### 3.8. Nursing Satisfaction

The patient satisfaction with humanized nursing in the therapy group was 97.80%, and the satisfaction with routine nursing in the control group was 26.67% (as displayed in Table 3). It was concluded that patient satisfaction in the therapy group was significantly higher than that in the control group, and the difference was statistically significant (*P* < 0.05).

## 4. Discussion

Sepsis is a systemic inflammatory response syndrome caused by bacteria and other pathogenic microorganisms invading the body. It is often secondary to various serious infections; it can lead to an imbalanced response of the patient's body to bacterial, fungal, viral, and parasitic infections, and cause multiple organ failure [15]. Severe sepsis is the severe stage of sepsis, which refers to the occurrence of one or more organ dysfunctions on the basis of sepsis, of which renal failure is one of the symptoms [16]. In the human body, it undertakes the functions of excreting waste, maintaining the body's acid-base balance, and adjusting ion balance. The failure of renal function will lead to the inability to remove toxins in the blood and the electrolyte imbalance of the body. Therefore, continuous blood purification therapy is applied to the treatment of patients with sepsis. In recent years, CRRT has been widely extended to emergency treatment of common critical illnesses, and has become one of the most important supportive measures in the treatment of various critical illnesses [17, 18]. Basic treatment methods can help patients recover to a certain extent, but for patients with severe sepsis, various functions of the body are seriously damaged, various organ failures, the patient's movement is limited, and the psychological pressure increases sharply. At the same time, continuous blood purification treatment will involve the extracorporeal circulation of blood. During this process, if the sterile state of the operating environment cannot be guaranteed, or the connection of equipment pipelines and filters is not tight, the patient may be reinfected, thereby aggravating the disease [6]. Therefore, adding certain nursing interventions can help patients control their condition, speed up their recovery, and bring some spiritual comfort to patients, thereby enhancing their confidence in overcoming the disease. This concept has also been confirmed from the experimental results. The APACHE-II scoring system is a scoring method for assessing disease severity in critically ill patients [19]. Patients with severe sepsis may experience abnormal changes in physiological indicators at any time due to organ failure, such as electrolyte imbalance, severe acidosis, arrhythmia, and the APACHE-II score will also change accordingly. On the 7th day and the 14th day of the experimental observation, the APACHE-II scores of the control group and the observation group all showed different degrees of decline. However, compared with the control group, the scores of the observation group decreased to a greater extent, which means that the electrolyte levels, body acid-base balance, and cardiac exercise of the patients recovered better under the nursing intervention. Patients with sepsis will experience hypoperfusion of various tissues and organs in the body due to hypoxia, anaerobic glycolysis, and finally, the accumulation of lactic acid, leading to metabolic and/or respiratory acidosis in patients [20]. Through the experiment, it was found that the lactic acid level in the observation group decreased more significantly than that in the control group, and the recovery of the patients' body temperature, respiration, heart rate, finger pulse oxygen saturation, and other indicators were also due to the control group.

The severity of cardiac insufficiency is closely related to brain natriuretic peptide (BNP) levels. When cardiac function declines, the natriuretic peptide system is activated, the cardiac load increases, and BNP release increases [21]. The levels of blood urea nitrogen and creatinine can reflect the renal function, and the improvement of serum brain natriuretic peptide, blood urea nitrogen, and creatinine in the observation group is better, which means that the recovery of renal function and cardiac function of patients under nursing intervention is more impressive. The uncontrolled expression of cytokines in patients with sepsis can cause cellular immune disorders, inflammatory responses, and secondary coagulation disorders. In severe infection, PCT is a more specific and sensitive serological indicator [22]. Researchers have found that PCT is involved in the sepsis response and has a certain correlation with inflammatory mediators. It can amplify the pathological process of sepsis and further aggravate the disease. It is the best marker for sepsis treatment and diagnosis [23]. In the experimental results, the levels of WBC, CRP, erythrocyte sedimentation rate, ESR, and PCT in the observation group and the control group decreased on the 7th and 14th days after treatment. Compared with the control group, the observation group decreased more significantly, indicating that the inflammation in the body was significantly improved. CD4+ is called helper T cells, CD8+ is called cytotoxic T cells, and its value can reflect the immune level of the body. The levels of CD4+ and CD4+/CD8+ in the nursing group showed an upward trend, and the levels of CD4+ and CD4+/CD8+ in the observation group were significantly higher than those in the control group, indicating that the recovery of the body's immune function under the nursing intervention was due to the control group. The final patient survival rate also improved with nursing intervention, as high as 71%. Under the nursing intervention, the patients' acceptance of treatment was higher and their attitude towards treatment was more positive, so the proportion of patients who gave up treatment due to physical or psychological reasons was also less than 5%. After professional medical means and monitoring, the phenomena of blood coagulation, abnormal body temperature, and vascular access obstruction are avoided. Therefore, the probability of lactic acid accumulation, abnormal body temperature, pipeline blockage, and coagulation disorder in the corresponding observation group was only 4.4%, which was significantly lower than that in the control group (15.6%). At the same time, humanized nursing has brought a certain positive effect on the physical and mental recovery of patients. The patients' satisfaction with personalized nursing was 97.80%, which was significantly higher than that of the control group, which was 26.67%.

## 5. Conclusion

Under the intervention of humanized nursing, the APACHE-II score, LAL, BUN, CRP, BNP, inflammatory factor levels, survival rate, and nursing satisfaction of the patients who implemented CBP therapy were better than those of the control group. Therefore, humanized nursing combined with CBP can not only meet the needs of patients psychologically but also avoid the occurrence of complications. In addition, timely monitoring and scientific nursing can reduce the inflammation level of the patient and restore body function faster, which was a more efficient treatment method for the patient's disease recovery.

## Figures and Tables

**Figure 1:** Specific operations of CBP.

**Figure 2:** Flow chart of experiment process.

**Figure 3:** Comparison of general conditions of patients with severe sepsis in different treatment stages. *Note*: ^*∗*^ meant *P* < 0.05 against the control group.

**Figure 4:** Comparison of APACHE-II scores of severe sepsis patients at different treatment stages. *Note*: ^*∗*^ meant *P* < 0.05 against the control group.

**Figure 5:** Comparison of BUN, CRP, and BNP of patients at different stages. *Note*: figures (a), (b), and (c) showed the comparison of BNP, BUN, and CRP, respectively. ^*∗*^ meant *P* < 0.05 against the control group.

**Figure 6:** Comparison of inflammatory indicators (WBC, CRP, ESR, PCT, and TNF-*α*). *Note*: figures (a)∼(e) showed the comparison of WBC, CRP, ESR, PCT, and TNF-*α*, respectively. ^*∗*^ meant *P* < 0.05 against the control group.

**Figure 7:** Comparison of CD4+, CD8+, and CD4+/CD8+. *Note*: figures (a), (b), and (c) illustrated the comparison of CD4+, CD8+, and CD4+/CD8+, respectively. ^*∗*^ meant *P* < 0.05 against the control group.

**Figure 8:** Comparison of proportions of survival, mortality, and giving treatment up.

**Table 1:** Comparison of the prognosis of the two groups of patients.

Group	Prognosis		
	Survival	Mortality	Other
Control group (45 cases)	21 (47%)^*∗*^	19 (42%)	5 (11%)
Therapy group (45 cases)	32 (71%)^*∗*^	11 (24%)	2 (5%)

*Note*. ^*∗*^ meant *P* < 0.05 against the control group.

**Table 2:** Comparison of the incidence of complications between the two groups of patients.

Group	Lactic acid accumulation	Abnormal body temperature	Pipeline blockage	Coagulation disorder	Incidence of complications
Control group (45 cases)	2	2	1	2	15.60%
Observation group (45 cases)	0	1	0	1	4.40%^*∗*^

*Note*. “^*∗*^” indicated that compared with the control group, the difference was statistically significant (*P* < 0.05).

**Table 3:** Satisfaction on humanized nursing and routine nursing.

Group	Very satisfied	Satisfied	General	Satisfaction
Control group (45 cases)	2	10	33	26.67%
Therapy group (45 cases)	26	18	1	97.80%
*X* ^2^	5.923	0.545	17.612	17.455
*P*	0.012	0.435	0.001	0

## Data Availability

The data used to support the findings of this study are included within the article.
